The article "Processing and Characterization of Novel Bio-Waste Hybrid Brick Composites for Pollution Control" was retracted in 2023. Reasons: signs of a paper mill; compromised peer review; unreliable results or conclusions.

# Processing and Characterization of Novel Bio-Waste Hybrid Brick Composites for Pollution Control

**DOI:** 10.1155/2022/3127135

**Published:** 2022-07-21

**Authors:** Naresh Kumar, Piyush Gaur, S. Kaliappan, L. Natrayan, S. Socrates, Pravin P. Patil, Subash Thanappan

**Affiliations:** ^1^Mechanical Engineering Department, Green Hills Engineering College, Solan 173229, India; ^2^School of Aeronautical Science, Hindustan Institute of Technology and Science, Padur, Chennai 603103, Tamil Nadu, India; ^3^Department of Mechanical Engineering, Velammal Institute of Technology, Chennai 601204, Tamil Nadu, India; ^4^Department of Mechanical Engineering, Saveetha School of Engineering, SIMATS, Chennai 602105, Tamil Nadu, India; ^5^Department of Mechanical Engineering, Graphic Era Deemed to be University, Bell Road, Clement Town, Dehradun 248002, Uttarakhand, India; ^6^Department of Civil Engineering, Ambo University, Ambo, Ethiopia

## Abstract

The main focus of this research is to enhance the use of eco-friendly materials these days. The current materials used in building construction are chemical-based and are harmful to humans and the environment. This research work has developed a new type of hybrid brick by using natural fibres and waste materials. This research focuses on fabricating novel bricks reinforced with different percentages of coconut waste fibre, wheat straw fibre, waste wood animal dung ash, gypsum, sand, and cement. The fabricated novel brick's physical, mechanical, chemical, acoustic, and heat-absorbing properties were evaluated.

## 1. Introduction

The recent building materials are costly and are not eco-friendly. These building materials have been utilized since ancient times [1]. Romans have suggested using natural fibres to stop the shrinkage of nonbacked bricks [2]. The use of natural fibre maintains dimension stability [3]. The natural fibre base material has many advantages: easy availability, low cost, fast regrowing, easy shape, and high strength [4]. The recent materials used to construct bricks have many harmful effects [5]. These materials are not eco-friendly and cause many diseases. The materials are chemical and cause diseases such as lung cancer, breathing problems, allergy, and skin problems [6]. The bricks produced by these materials absorb heat and cold and show less thermal stability. These materials are not so good in less absorbing [7]. Various factories produce lime sludge, including paper mills, sugar mills, marble mills, and fertilizer. All sludge has certain harmful constituents/contaminants from the manufacturing process; for example, paper mill sludge contains up to 2% free alkalis [8]. These harmful chemicals prevent cement and associated construction materials from being used in bulk. The plain mortar of ratio 1:5 resulted in an overall consumption of fly-ash of about 75% and a cost savings of around 58% (cement: sand) [9]. Using fly-ash in a mortar designed by weight saves 50%–60% of the cost, whereas using it in a mortar designed by volume saves 9%–16% of the cost. The fly-ash mortar blend 1 : 1 : 5 (cement: fly-ash: sand) by weight, on the other hand, uses around 20% cement and consumes 20% less fly-ash overall [10].

The article "Processing and Characterization of Novel Bio-Waste Hybrid Brick Composites for Pollution Control" was retracted in 2023. Reasons: signs of a paper mill; compromised peer review; unreliable results or conclusions.

Chemical materials have been replaced with eco-friendly and waste materials to produce novel-type bricks. Coconut fibre is utilized because it is a natural waste fibre with good mechanical properties [11]. Wheat fibre waste material is utilized because the handling of wheat-based waste fibre has become a serious challenge for India and worldwide. These materials are also caused to produce pollution to the environment. These materials are associated with serious safety issues on railways and highways [12]. Every year, thousands of tons of wheat fibre are burnt openly to dispose of it in Punjab, Haryana, and different parts of India and the world. In this paper, wheat fibre has been utilized in the bricks to find the solution to this waste material [13]. The wood waste material is mostly used to burn.Waste Concrete Bricks were combined with cotton (1 to 5%), recycled paper mill waste (89% to 85%), and cement (10%). Owing to tiny air pockets inside paper waste, the bricks produced were a little light (half the weight of traditional clay brick). A homogenizer and a hand-operated hydraulic press were both planned and built. They suggested a two-stage press procedure to maintain the smoothness of the surface during drying [14]. The mechanism of strength production was a typical pozzolanic reaction. But, due to the cellulosic nature of cotton waste, high water absorption has also been noted. Crushed rock flour will substitute up to 40% of sand, but as the amount of sand replaced by rock flour increases, the workability decreases slightly [15]. The addition of nano-silica extracted from olivine increases the financial attractiveness of concrete and reduces the final product's CO_2_ footprints [16]. Coal combustion by-products are generated by mixing fly-ash and cement in civil construction schemes, forming bricks, and using them as a road pavement material and soil enrichment medium for plant growth [17]. Increased amounts of natural sand were substituted for ground waste glass, resulting in a significant improvement in compressive ability. In this paper, wood waste material has been utilized to develop bricks because it is compatible with cement [18]. Cow dung has good thermal and acoustic properties and also has good binding properties, so cow dung has also been used in these novel bricks [19]. Second, animal dug wastage was used because it is also used to increase thermal stability.

The article "Processing and Characterization of Novel Bio-Waste Hybrid Brick Composites for Pollution Control" was retracted in 2023. Reasons: signs of a paper mill; compromised peer review; unreliable results or conclusions.

A novel of this research work is to fabricate the novel bricks reinforced with different percentages of coconut waste fibre, wheat straw fibre, waste wood, animal dung ash, gypsum, sand, and cement. Fabricated novel brick's physical, mechanical, chemical, acoustic, and heat-absorbing properties were evaluated.

## 2. Materials and Methods

### 2.1. Composite Fabrication

The coconut fibres were purchased from a vegetable shop, and after that, the fibres were removed from the coconut's upper surface. The unwanted material was removed from the surface of the coconut by hand [20]. After that, the chemical treatment was given to the fibres to remove impurities [21]. The ash content received after burning the sissoo wood and impurities were removed with the help of a stainer. The waste wood particles were collected from the carpenter shop. Then, dried cow dung was collected from the village and converted into very small particles [22]. All these materials were mixed with cement and sand.  Table 1 shows the compositional details of the materials [23]. For proper mixing of these materials, all these materials were mixed using a plough machine [24]. The composition of the hybrid brick is shown in Figure 1. The experiments were performed according to the Standards BS 3921 : 1985 and MS 76 : 1972 [25]. The moulded size was 225 × 162 × 68 mm cubes. Composite fabrication details are shown in Table 2.

Based on the findings and experimental methodology, it can be inferred that concrete manufactured with over-burnt concrete waste aggregate and brick ballast performed better than concrete made with natural aggregate collected from local supplies. Where natural aggregates are not readily available, high concrete strength is not needed. It is recommended that broken over-burned bricks be used as coarse aggregate in structural concrete.

### 2.2. Physico-mechanical, Acoustic, Chemical, and Thermal Properties

A universal testing machine (UTM) measured mechanical properties such as tensile strength and tensile modulus [26]. The impact energy test was performed on the Charpy impact testing machine. Flexural strength and flexural modulus were performed on a pendulum testing machine (ASTMED790 standard). The density was measured using a Wenser weighing machine [27]. To determine the porosity of newly developed bricks samples, the samples were dipped into the water. The water absorption test brick was soaked in water for 24 hours. Water absorption = weight of brick before the dipping- the weight of brick after dipping. A crushing test was performed to determine the crushing strength on a compression testing machine with ASTM C1314-14 standard [28]. A heat absorption test was performed to find the heat absorbed by the material [29]. The brick was put into the muffle furnace for 2 hours at 60°C, and after the brick was removed, the temperature was noticed at the same time after 15 minutes. Similarly, the bricks were held at −5°C and the temperature was noted at the same time as well after 15 minutes. The newly developed bricks were put into the furnace for 8 hours at 1000°C [30]. The shear strength bond test was used to find the bound between three bricks [31]. A small size of 4 feet and 4 feet of small space such as a room was developed with BA-1, BA-2, BA-3, and BA-4 samples to record the sound using a sound level meter [32].

The article "Processing and Characterization of Novel Bio-Waste Hybrid Brick Composites for Pollution Control" was retracted in 2023. Reasons: signs of a paper mill; compromised peer review; unreliable results or conclusions.

## 3. Results & Discussion

### 3.1. Chemical, Physical, Mechanical, and Tri-Biological Characterization of Coconut/Wheat Straw-Based Bricks

It has been investigated that as the percentage of coconut fibre and wheat straw fibre in the brick reinforced material increases, the brick's shear bond strength is decreases [33]. The BA-1-based brick has shown the best shear bond strength (0.3 MPa). The BA-1-based brick has shown the maximum crushing strength (3.05 N/mm^2^). The crushing strength will decrease because the high dense filler ash and high bounding cement have been replaced by the low wt natural fibre [34]. The BA-1- and BA-2-based bricks have shown minimum porosity (7% and 9%, respectively); as the percentage of organic fibre in the brick material increases, the porosity will increase. In opposite porosity, density shows its minimum value for the BA-4 (1450 kg/m^3^) organic fibre-based brick. The BA-4 composite shows the highest density value (1700 kg/m^3^).

The level of water absorption will increase as the percentage of coconut fibre and wheat straw fibre in the brick material increases. BA-1 has shown minimum water absorption (9%). Increased water absorption with an increasing percentage of coconut fibre and wheat straw is because high-dense weight ash cement and sand have been replaced by the low-weight organic fibre [35]. The BA-1 brick has shown minimum heat swelling (3%). At a temperature of 150°C, the swelling increases the coconut fibre and wheat straw fibre in the brick material. The tensile strength of the brick shows maximum strength for BA-2 brick (1.5 MPa). The tensile strength and shear strength increase because coconut and wheat straw fibres act as binders in the brick composite material and increase the bonding strength. The impact strength has shown its highest value for BA-3 bricks (0.57 N-m), which might increase the fibre's work as a binder and increase the impact strength of the brick. The BA-2 brick has shown the highest value of the modulus of elasticity (16.42 MPa), and BA-4 has shown a minimum modulus of elasticity (14 MPa). The ash percentage has shown a minimum value for the BA-1-based brick. The flexural strength was investigated for BA-1 (0.48). The change in brick volume was recorded as a minimum for BA-1 (.05%).  Table 3 shows the characterizations of cocco and waste wheat straw bricks [36].

The article "Processing and Characterization of Novel Bio-Waste Hybrid Brick Composites for Pollution Control" was retracted in 2023. Reasons: signs of a paper mill; compromised peer review; unreliable results or conclusions.

### 3.2. Heat-Absorbing Properties of Specimens

During the heat-absorbing test, it has been investigated that the BA-3 and BA-4 bricks absorb less heat, as shown in Figure 2. The BA-4 brick has shown a minimum heat-absorbing capacity (14°C), and BA-1 has maximum heat-absorbing capacity (18°C). In the heat-absorbing test, at 0°C, the BA-4 brick has shown a minimum value of heat-absorbing (11°C), and the BA-4 brick shows maximum temperature (11°C). Increasing the percentage of wheat fibre, coco fibre with ash, and dug in the composites, the heat-absorbing capacity (high and low temperatures) shows less effect because these do not absorb heat [37].

The water absorption capacity ranged from 12.6% to 29.20%. As opposed to conventional clay bricks, all bricks produced in this study had a 30% improvement in fire resistance and were more durable in terms of corrosion resistance and weight gain [38].

### 3.3. Heat-Dissipating Capacity of Brick

During the heat-dissipating test, it has been investigated that the BA-3 and BA-4 bricks absorb less heat with different temperatures (20°C, 30°C, 40°C, 50°C, and 60°C) and different time variations (5, 10, 15, and 20 minutes) among all newly developed samples, as shown in Figure 3. During the tests, it was investigated that BA-3 and BA-4 brick samples showed maximum heat dissipation after 20 minutes. All newly developed samples BA-1, BA-2, BA-3, and BA-4 show minimum heat dissipation after 5 minutes of time and maximum heat dissipate at 20 minutes [39].  Figure 4 shows the temperature loss with the time of the BA-2 brick composites.  Figure 5 shows the temperature loss with a time of the BA-3 bricks composites [40]. Tables 4 and 5 show the heat-absorbing capacity at different temperatures. Temperature loss with the time of BA-4 brick composites is shown in Figure 6. The heat dissipating capacity with different temperatures and different times for the BA-1 sample is shown in Table 6.

Natural coarse aggregate can be replaced with recycled clay brick aggregate. Recycled clay-brick aggregate concrete can achieve enough strength and can be used to make medium- and low-strength concrete. This paper looks at clay brick waste as a partial cement and concrete substitute material. The performance of mortar and concrete in mechanical and durability-related properties has been discussed [41].

The article "Processing and Characterization of Novel Bio-Waste Hybrid Brick Composites for Pollution Control" was retracted in 2023. Reasons: signs of a paper mill; compromised peer review; unreliable results or conclusions.

Table 7 shows the heat-dissipating capacity with different temperatures and different times for the BA-2 samples. The heat dissipating capacity with temperatures and different times for the BA-3 samples is shown in Table 8. The heat dissipating capacity with different temperatures and different times for the BA-4 samples is shown in Table 9.

The freshly moulded green bricks, which contain approximately 25% moisture by weight, are left out in the open; they are first dispersed on the field and then piled in layers to gradually dry to a moisture content of 3%–15%. The bricks are then set on fire, the mechanical moisture is removed up to a firing temperature of less than 200 degree Celsius (°C), the inherent carbonaceous matter is burned from 350 to 700 degree Celsius (°C), endothermic decomposition of clay molecules occurs from 400 to 600 degree Celsius, and chemically combined water is evaporated from 400 to 600 degree Celsius [42].

### 3.4. Sound-Absorbing Capacity of Specimens

During the sound-absorbing tests, it has been investigated that as the percentage of coconut fibre and wheat waste fibre in the newly developed composition increases, the sound level decreases, while the sound absorption capacity of the bricks increases.  Table 10 shows the minimum weighted normalized sound level difference (Dn, w) for building walls according to DL 129/2002. The BA-1 based brick shows the highest sound, and B-4 based brick shows the lowest [43]. The cause of this is all materials such as wheat waste fibre, coconut fibre, wood, and dung are sound-absorbing materials [44], with an increased percentage of natural fibres and waste fibre sound-absorbing capacity increase shown in Figure 7.

The Portuguese code allows for a 3 dB margin to take measurement uncertainties into account.

## 4. Conclusion

Novel bricks reinforced with different percentages of coconut waste fibre, wheat straw fibre, waste wood, animal dung ash, gypsum, sand, and cement were fabricated successfully. The following conclusions were drawn:

- The BA-1-based brick has shown maximum compressive strength (3.05 N/mm^2^) while BA-4-based brick has shown the lowest value of brick strength (2.30 N/mm^2^).
- Porosity has been noticed to increase the percentage of coconut and wheat waste fibre in the new composition. The BA-1-based brick has shown minimum porosity (7%). Ash content was found to be minimum for the BA-1-based brick.
- The water absorption capacity was increased with an increased percentage of coconut waste fibre and wheat waste fibre in the mould. The BA-1-based brick has shown minimum water absorption and minimum density (1450 kg/m^3^). The BA-4 brick has shown minimum heat swelling (3%).
- The impact was maximum for BA-3-based composites (4.90 N-m). The maximum shear bonding strength was found for the BA-1-based brick (0.3 MPa).
- The sound test has investigated that BA-3- and BA-4-based bricks absorb maximum sound and show better acoustic properties. The test found that BA-3- and BA-4-based bricks absorb minimum heat and dissipate maximum heat in heat absorption and dissipation. The tensile strength was maximum for the BA-3-based brick (1.5 MPa) while flexural bond strength and modulus of elasticity have shown their maximum value for BA-1-based bricks.

The article "Processing and Characterization of Novel Bio-Waste Hybrid Brick Composites for Pollution Control" was retracted in 2023. Reasons: signs of a paper mill; compromised peer review; unreliable results or conclusions.

This paper has shown that new green building bricks have good physical, mechanical, acoustic, and thermal properties.

## Figures and Tables

**Figure 1:** (a) Newly developed brick sample (b) Crushing test in a compression machine.

**Figure 2:** Heat-absorbing capacity at variant temperatures.

**Figure 3:** Temperature loss with the time of BA-1 brick composites.

**Figure 4:** Temperature loss with the time of BA-2 bricks composites.

**Figure 5:** Temperature loss with the time of BA-3 bricks composites.

**Figure 6:** Temperature loss with the time of the BA-4 bricks composites.

**Figure 7:** Sound values with different developed samples.

**Table 1:** Compositional details of materials.

Fabrication of the composites					
S. No	Name of sample	BA-1	BA-2	BA-3	BA-4
1	Coconut waste fibres	5	10	15	20
2.	Waste wood	5	5	5	5
3	Ash	15	15	15	15
4	Waste wheat straw	5	10	15	20
5	Animal dug	10	10	10	10
6	Sand	25	20	15	10
7	Cement	30	25	20	15
8	Gypsm	5	5	5	5

**Table 2:** Composites fabrication detail.

Condition	Process
Mixing condition	The materials used are as follows: coconut waste fibre, wood, wheat straw, animal drugs, sand, cement, and gypsum.
	Coconut waste fibre, wood, wheat straw, and animal dung were mixed for the first ten mins
	After that, cement, sand, and water were mixed with the ingredients and mixed for another ten minutes.

Moulding conditions	The mixed material was poured into the mould and levelled, and kept in the mould for two days.

Dry condition	The newly developed bricks were held in the environmental atmosphere, and water was provided daily to avoid the cracks and increase the strength
	After 6 days, the developed bricks were put in the muffle furnace at 60°c to remove the moisture for 8 hours.

**Table 3:** Characterizations of cocco and waste wheat straw bricks (mechanical, physical, and chemical).

Properties	Standard used	BA-1	BA-2	BA-3	BA-4
% Porosity	ASTM C 29/C 29M-97	7	9	11	14
% Ash content	ASTMD570-98	63	67	60	75
% Water Absorption	IS 1077 : 1992	9	9.5	10	11
Density [kg/m^3^]	IS 2185-1 (2005)	1700	1620	1510	1450
Crushing strength (N/mm^2^)	ASTM C1314-14	3.05	2.90	2.60	2.30
% Heat swelling	SAE J 160 JNU80	3	3.8	5	7
Impact Energy (N-m)	ASTM D256	0.47	0.53	0.57	0.490
Shear bound strength (MPa)	RILEM TC 127-MS	0.3	0.29	0.27	0.25
Tensile strength (MPa)	ASTM C1314-14	1.4	1.5	1.0	0.9
Flexural bound strength (MPa)	ASTM E518	0.48	0.42	0.39	0.35
Modulus of elasticity (MPa)	ASTM C1314-14	16.42	15.6	15	14

The article "Processing and Characterization of Novel Bio-Waste Hybrid Brick Composites for Pollution Control" was retracted in 2023. Reasons: signs of a paper mill; compromised peer review; unreliable results or conclusions.

**Table 4:** Heat-absorbing capacity at different temperatures.

Temperature	BA-1	BA-2	BA-3	BA-4
20°C	18	16	15	14
30°C	25	23	20	17
40°C	35	30	25	22
50°C	38	35	28	26
60°C	45	40	31	28

**Table 5:** Heat-absorbing capacity at low temperature[0°C].

Temperature	BA-1	BA-2	BA-3	BA-4
0°C	6	7	10	11

**Table 6:** Heat dissipating capacity with different temperatures and different times for the BA-1 samples.

BA-1				
Temperature	5 minutes	10 minutes	15 minutes	20 minutes
20°C	18	16	14	14
30°C	24	20	16	14
40°C	36	30	24	22
50°C	45	40	26	24
60°C	52	45	28	26

**Table 7:** Heat dissipating capacity with different temperatures and different times for the BA-2 samples.

BA-2				
Temperature	5 minutes	10 minutes	15 minutes	20 minutes
20°C	17	15	14.7	14
30°C	23	19	15	16
40°C	34	28	22	20
50°C	43	38	24	22
60°C	52	43	26	24

**Table 8:** Heat dissipating capacity with different temperatures and different times for the BA-3 samples.

BA-3				
Temperature	5 minutes	10 minutes	15 minutes	20 minutes
20°C	16.6	15.5	14.7	14
30°C	22.5	18.6	14.8	14.6
40°C	33.8	27.6	21.6	19.8
50°C	42.4	37.4	23.6	21.6
60°C	51	44	24.6	23.4

**Table 9:** Heat dissipating capacity with different temperatures and different times for the BA-4 samples.

BA-3				
Temperature	5 minutes	10 minutes	15 minutes	20 minutes
20°C	16	15	14.4	14
30°C	22	18	14.4	14.2
40°C	33	26	20	18.4
50°C	41	36	22.4	21.6
60°C	46	40	22	21

**Table 10:** Minimum weighted normalized sound level difference (Dn, w) for building walls according to (DL 129/2002).

Sample	Dn, w ≥ (dB)	Dn, w—3*∗*≥ (dB)
BA-1	42	38
BA-2	40	37
BA-3	38	35
BA-4	35	32

## Data Availability

The data used to support the findings of this study are included in the article. Should further data or information be required, these are available from the corresponding author upon request.

## References

[1] Viegi G., Scognamiglio A., Baldacci S., Pistelli F., Carrozzi L. (2001). Epidemiology of chronic obstructive pulmonary disease. *COPD) Respiration*.

[2] Oleru U. G. (1984). Pulmonary function and symptoms of Nigerian workers exposed to cement dust. *Environmental Research*.

[3] Al-Neaimi Y. I., Gomes J., Lloyd O. L. (2001). Respiratory illnesses and ventilatory function among workers at a cement factory in a rapidly developing country. *Occupational Medicine*.

The article "Processing and Characterization of Novel Bio-Waste Hybrid Brick Composites for Pollution Control" was retracted in 2023. Reasons: signs of a paper mill; compromised peer review; unreliable results or conclusions.

[4] Mirzaee R., Kebriaei A., Hashemi S. R., Sadeghi M., Shahrakipour M. (2008). Effects of exposure to Portland cement dust on lung function in Portland cement factory workers in Khash, Iran. *Iranian Journal of Environmental Health Science & Engineering*.

[5] Neghab M., Choobineh A. (2007). Work related respiratory symptoms and ventilatory disorders among employees of a cement industry in Shiraz, Iran. *Journal of Occupational Health*.

[6] Zeleke Z. K., Moen B. E., Bratveit M. (2011). Lung function reduction and chronic respiratory symptoms among workers in the cement industry: a follow up study. *BMC Pulmonary Medicine*.

[7] Thepaksorn P., Pongpanich S., Siriwong W., Chapman R. S., Taneepanichskul S. (2013). Respiratory symptoms and patterns of pulmonary dysfunction among roofing fiber cement workers in the south of Thailand. *Journal of Occupational Health*.

[8] Olotuah A. O. (2002). Recourse to earth for low-cost housing in Nigeria. *Building and Environment*.

[9] Bejaxhin A. B. H., Paulraj G., Aravind S. (2020). Influence of TiN/AlCrN electrode coatings on surface integrity, removal rates and machining time of EDM with optimized outcomes. *Materials Today Proceedings*.

[10] Lakshmipathy R., Sarada N. C. (2015). A fixed bed column study for the removal of Pb2+ ions by Watermelon rind. *Environmental Sciences: Water Research & Technology*.

[11] Veeman D., Sai M. S., Sureshkumar P. (2021). Additive manufacturing of biopolymers for tissue engineering and regenerative medicine: an overview, potential applications, advancements, and trends. *International Journal of Polymer Science*.

[12] Quagliarini E., Lenci S., Iorio M. (2010). Mechanical properties of adobe walls in a Roman Republican domus at Suasa. *Journal of Cultural Heritage*.

[13] Quagliarini E., Lenci S. (2010). The influence of natural stabilizers and natural fibres on the mechanical properties of ancient Roman adobe bricks. *Journal of Cultural Heritage*.

[14] Russ W., Mörtel H., Meyer-Pittroff R. (2005). Application of spent grains to increase porosity in bricks. *Construction and Building Materials*.

[15] Suryanarayanan R., Sridhar V. G., Natrayan L. (2021). Improvement on mechanical properties of submerged friction stir joining of dissimilar tailor welded aluminum blanks. *Advances in Materials Science and Engineering*.

[16] Lakshmipathy R., Sarada N. C. (2016). Methylene blue adsorption onto native watermelon rind: batch and fixed bed column studies. *Desalination and Water Treatment*.

[17] Bovas Herbert Bejaxhin A., Paulraj G., Jayaprakash G., Vijayan V. (2021). Measurement of roughness on hardened D-3 steel and wear of coated tool inserts. *Transactions of the Institute of Measurement and Control*.

The article "Processing and Characterization of Novel Bio-Waste Hybrid Brick Composites for Pollution Control" was retracted in 2023. Reasons: signs of a paper mill; compromised peer review; unreliable results or conclusions.

[18] Yetgin Ş., Çavdar O., Çavdar A. (2008). The effects of the fiber contents on the mechanic properties of the adobes. *Construction and Building Materials*.

[19] Binici H., Aksogan O., Bakbak D., Kaplan H., Isik B. (2009). Sound insulation of fibre reinforced mud brick walls. *Construction and Building Materials*.

[20] Ali S., Kumar N., Thakur V., Chau K. W., Kumar M. (2022). Coconut waste fiber used as brake pad reinforcement polymer composite and compared to standard kevlar-based brake pads to produce an asbestos free brake friction material. https://onlinelibrary.wiley.com/doi/10.1002/pc.26472?af=R.

[21] Romasanta R. R., Sander B. O., Gaihre Y. K. (2017). How does burning of rice straw affect CH4 and N2O emissions? A comparative experiment of different on-field straw management practices. *Agriculture, Ecosystems & Environment*.

[22] Devarajan Y., Nagappan B., Choubey G., Vellaiyan S., Mehar K. (2021). Renewable pathway and twin fueling approach on ignition analysis of a dual-fuelled compression ignition engine. *Energy & Fuels*.

[23] Lakshmipathy R., Sarada N. C. (2016). Metal ion free watermelon (*Citrullus lanatus*) rind as adsorbent for the removal of lead and copper ions from aqueous solution. *Desalination and Water Treatment*.

[24] Zhang Y., Zang G.-Q., Tang Z.-H., Chen X.-H., Yu Y.-S. (2014). Burning straw, air pollution, and respiratory infections in China. *American Journal of Infection Control*.

[25] Korjenic A., Zach J., Hroudová J. (2016). The use of insulating materials based on natural fibers in combination with plant facades in building constructions. *Energy and Buildings*.

[26] John V. M., Cincotto M. A., Sjöström C., Agopyan V., Oliveira C. T. A. (2005). Durability of slag mortar reinforced with coconut fibre. *Cement and Concrete Composites*.

[27] Natrayan L., Merneedi A. (2021). Experimental investigation on wear behaviour of bio-waste reinforced fusion fiber composite laminate under various conditions. *Materials Today Proceedings*.

[28] Devarajan Y., Choubey G., Mehar K. (2019). Ignition analysis on neat alcohols and biodiesel blends propelled research compression ignition engine. *Energy Sources, Part A: Recovery, Utilization, and Environmental Effects*.

[29] Zhou X.-Y., Zheng F., Li H.-G., Lu C.-L. (2010). An environment-friendly thermal insulation material from cotton stalk fibers. *Energy and Buildings*.

[30] Bołtryk M., Anna K., Pawluczuk E. (2020). Cement composites with wood waste—design, features, and proposal of application. *Aci Materials*.

The article "Processing and Characterization of Novel Bio-Waste Hybrid Brick Composites for Pollution Control" was retracted in 2023. Reasons: signs of a paper mill; compromised peer review; unreliable results or conclusions.

[31] Katale D. P., Kamara V. S., Adedeji A. A. (2014). Investigation on the Use of Clayey Soil Mixed with Cow Dung to Produce Sustainable Bricks. https://scialert.net/fulltext/?doi=tasr.2014.406.424.

[32] Ali N., Zainal N. A., Burhanudin M. K. (2016). Physical and mechanical properties of compressed earth brick (CEB) containing sugarcane bagasse ash. *MATEC Web of Conferences*.

[33] Ullah Qureshi A. (2020). *Compressive Strength of Fly Ash Brick with Lime Gypsum & Quarry Dust*.

[34] Akinyele J. O., Igba U. T., Ayorinde T. O., Jimoh P. O. (2020). Structural efficiency of burnt clay bricks containing waste crushed glass and polypropylene granules. *Case Studies in Construction Materials*.

[35] Yogeshwaran S., Natrayan L., Rajaraman S., Parthasarathi S., Nestro S. (2021). Experimental investigation on mechanical properties of epoxy/graphene/fish scale and fermented spinach hybrid bio composite by hand lay-up technique. *Materials Today Proceedings*.

[36] Devarajan Y., Munuswamy D. B., Nalla B. T., Choubey G., Mishra R., Vellaiyan S. (2022). Experimental analysis of Sterculia foetida biodiesel and butanol blends as a renewable and eco-friendly fuel. *Industrial Crops and Products*.

[37] Shakir A., Naganathan S., Mustapha K. N. (2013). Development of Bricks from waste material, 2013; A review paper Australian. *Journal of Basic & Applied Sciences*.

[38] Kumar N., Singh T., Grewal J. S., Patnaik A., Fekete G. (2019). A novel hybrid AHP-SAW approach for optimal selection of natural fiber reinforced non-asbestos organic brake friction compositesfiber reinforced non-asbestos organic brake friction composites. *Materials Research Express*.

[39] Kazmi S. M. S., Munir M. J., Wu Y. F., Hanif A., Patnaikuni I. (2018). Thermal performance evaluation of eco-friendly bricks incorporating waste glass sludge. *Journal of Cleaner Production*.

[40] Madani H., Ramezanianpour A. A., Shahbazinia M., Ahmadi E. (2020). Geopolymer bricks made from less active waste materials. *Construction and Building Materials*.

[41] Priyadarshini M., Giri J. P., Patnaik M. (2021). Variability in the compressive strength of non-conventional bricks containing agro and industrial waste. *Case Studies in Construction Materials*.

[42] dos Reis G. S., Cazacliu B. G., Cothenet A. (2020). Fabrication, microstructure, and properties of fired clay bricks using construction and demolition waste sludge as the main additive. *Journal of Cleaner Production*.

[43] Lalzarliana Paihte P., Lalngaihawma A. C., Saini G. (2019). Recycled Aggregate filled waste plastic bottles as a replacement of bricks. *Materials Today Proceedings*.

[44] Maza-Ignacio O. T., Jiménez-Quero V. G., Guerrero-Paz J., Montes-García P. (2020). Recycling untreated sugarcane bagasse ash and industrial wastes for the preparation of resistant, lightweight and ecological fired bricks. *Construction and Building Materials*.

